# *Crocus sativus* L. (Saffron) Stigma Aqueous Extract Induces Apoptosis in Alveolar Human Lung Cancer Cells through Caspase-Dependent Pathways Activation

**DOI:** 10.1155/2013/417928

**Published:** 2013-10-29

**Authors:** Saeed Samarghandian, Abasalt Borji, Seyed Kazem Farahmand, Reza Afshari, Saeideh Davoodi

**Affiliations:** ^1^Department of Basic Medical Sciences, Neyshabur Faculty of Medicine, Neyshabur, Iran; ^2^Health Strategic Research Center, Neyshabur Faculty of Medicine, Neyshabur, Iran; ^3^Medical Toxicology Research Centre, Mashhad University of Medical Sciences, Mashhad, Iran; ^4^Immunology Research Center, Bu-Ali Research Institute, Mashhad University of Medical Sciences, Mashhad, Iran

## Abstract

Worldwide, lung cancer is the most common form of cancer. Saffron has been used in folk medicine for centuries. We investigated the potential of saffron to induce cytotoxic and apoptotic effects in lung cancer cells (A549). We also examined the caspase-dependent pathways activation of saffron-induced apoptosis against the A549 cells. A549 cells were incubated with different concentrations of saffron extract; then cell morphological changes, cell viability, and apoptosis were determined by the normal invertmicroscope, MTT assay, Annexin V and propidium iodide, and flow cytometric analysis, respectively. Activated caspases were detected by treatment of saffron in lung cancer cells using fluorescein-labeled inhibitors of polycaspases. The proliferation of the A549 cells were decreased after treatment with saffron in a dose- and time-dependent manner. The percentage of apoptotic cells increased with saffron concentrations. Saffron induced morphological changes, decreased percentage of viable cells, and induced apoptosis. Saffron could induce apoptosis in the A549 cells and activate caspase pathways. The levels of caspases involved in saffron-induced apoptosis in the A549 cells indicating caspase-dependent pathway were induced by saffron. The anticancer activity of the aqueous extract of saffron could be attributed partly to its inhibition of the cell proliferation and induction of apoptosis in cancer cells through caspase-dependent pathways activation.

## 1. Introduction

Lung cancer is the leading cause of cancer-related death worldwide. Lung cancer is not only difficult to cure but it also tends to relapse easily; lung cancer also has a high incidence of recurrence [1, 2]. Therefore, the development of novel approaches and effective anticancer strategies is critically needed for prolonged survival of lung cancer and early being pursued [3]. Lung cancers are classified into the two main histological groups of lung cancer including non-small cell lung cancer (NSCLC, 85%) and small cell lung cancer (SCLC, 15%). It should be mentioned that the carcinomic human alveolar basal epithelial cell (A549) is the non-small cell lung cancer and the most common and widely studied cell line in lung cancer [4].

Some cancer chemotherapeutic agents can abate or reverse cancer development and/or progression. As an important source, plants may produce potential chemopreventive or chemotherapeutic agents. As a part of an effort to evaluate the newly emerging drugs for lung cancer, we studied the role of saffron on non-small cell lung cancer. 

Saffron is the dried stigma of the flowers of saffron (*Crocus sativus* L., Iridaceae). In addition to being a widely used food additive, saffron is used in the traditional medicine for vomiting, spasm, asthma, bronchitis, fever, colds, cardiovascular disorders, and also cancer [5–8]. It has been showed that saffron extracts exert antitumor, [9] free radical scavenging, hypolipemic [10], and anticonvulsant activities, [11] as well as improving learning and memory [12]. However, the molecular mechanism for the potent effect of saffron has not been yet clarified. 

Apoptosis is characterized by particular morphological changes, including plasma membrane bleb, cell shrinkage, depolarization of mitochondria, chromatin condensation, and DNA fragmentation [13]. The relationship between apoptosis and cancer has been a recent focus. Apoptosis provides a number of useful clues when generating effective therapies, and many chemotherapeutic agents exert their anticancer effects by inducing apoptosis in cancer cells [13]. Therefore, induction of apoptosis has become a principal mechanism by which anticancer therapy is effective [14].

In the present study, we examined the caspase-dependent pathways activation of saffron-induced apoptosis against A549 cell line. This study was designed to investigate the possible mechanisms of apoptosis induced by saffron in human alveolar adenocarcinoma (A549) cells. Therefore, at first, this study attempted to identify and confirm the cytotoxicity and apoptosis effects of saffron on the proliferation of the alveolar human lung cancer cell line, and then the current study tried to clarify the molecular pathways involved in apoptosis induced by saffron on the human lung cancer cells. We struggled to find whether caspase pathways were involved in the apoptotic effects of saffron on the A549 cells.

## 2. Materials and Methods

### 2.1. Chemicals and Reagents

3-(4,5-Dimethylthiazol-2-yl)-2,5-diphenyltetrazolium bromide (MTT) was purchased from Amerso (USA). Dulbecco's modified Eagle's medium (DMEM) was purchased from Gibco BRL (Grand Island, NY, USA). Annexin V/fluorescein isothiocyanate (FITC) was obtained from Invitrogen Corporation (Camarillo, CA, USA). Fetal bovine serum was purchased from PAA Laboratories GmbH, Austria.

Polycaspases FLICA (FAM-VAK-FMK) was purchased from ImmunoChemistry Technologies, LLC (ICT) (Minnesota, USA). 

### 2.2. Preparation of Aqueous Extract of Saffron

Saffron was supplied by SaharKhiz Co. (Mashhad, Iran) and was processed in the Pharmacological Research Center of Medicinal Plants. The part of *C. sativus* that is being used as additive and also as herbal medicine is the stigma. The stigma part of saffron was air-dried in the shade before extraction. After grinding, aqueous extract was prepared with 15 g of its ground petal stigma and 400 mL of distilled water in a Soxhlet extractor for 18 hours. The prepared extract was concentrated to 100 mL with a rotatory evaporator in low pressure and filtered through a 0.2 mm filter to be sterilized. The resultant solution was stored at 4°C to 8°C. Various concentrations of saffron (100, 200, 400, and 800 *μ*g/mL) and a control solution without saffron extract were prepared immediately and refrigerated before the experiments.

### 2.3. Cell Culture

The human non-small lung cancer cells (A549) and the human fetal lung fibroblast cell line (MRC-5) were obtained from Pasteur Institute (Tehran, Iran). The cells were grown either in 96-well tissue (TC) plate (NUNC, Wiesbaden, Germany) or in 25 cm^2^ TC flasks (NUNC, Wiesbaden, Germany), cultured in DMEM medium supplemented with 10% fetal bovine serum (FBS)(Gibco-Invitrogen), 100 U/mL of penicillin (Gibco-Invitrogen), and 100 *μ*g/mL streptomycin (Gibco-Invitrogen). A549 and MRC-5 cells were cultured in CO_2_ incubator MCO-17AI (Sanyo Electric Co., Ltd., Japan) at 37°C, in 95% humidified atmosphere enriched by 5% CO_2_ and subcultured every 3-4 days.

### 2.4. Cell Viability Assay

Cell viability was measured using the MTT assay, which is based on the conversion of MTT to formazan crystals by mitochondrial dehydrogenases [15]. Briefly, A549 and MRC-5 cells were plated at a density of 1 × 10^3^ cells/mL in 96-well plates and allowed to attach for 24 h to keep the log-phase growth at the time of drug treatment. Saffron at different concentrations (100, 200, 400, and 800 *μ*g/mL) was added to the wells for 24, 48 and 72 hours. After treatment with aqueous extract of saffron for 24, 48, and 72 h, 10 *μ*L MTT was added into each well. After 4 h incubation at 37°C, this solution was removed, and the produced formazan was solubilized in 100 *μ*L dimethyl sulfoxide (DMSO). Saffron extract has absorbance maxima around 550 nm. Absorbance was measured at 550 nm using an automated microplate reader (Bio-Rad 550). Cell viability was expressed as a percentage of the control culture value. The cytotoxic effects of saffron extract on cell lines (A549 and MRC-5) were expressed as IC_50_ value (the drug concentration reducing the absorbance of treated cells by 50% with respect to untreated cells). All experiments were carried out in triplicate.

### 2.5. Morphological Studies of Cell Lines Using the Inverted Microscope

Morphological studies using the normal inverted microscope were carried out to observe the morphological changes of cell death in the A549 cells elicited by the saffron extract. Different concentrations of saffron (200 and 400 *μ*g/mL) for 48 h were used for the morphological studies. The untreated cells served as the negative control. The morphological changes of the cells were observed under the normal inverted microscope after 48 h after-treatment.

### 2.6. Assessment of Apoptosis by Annexin V-FITC

Saffron has an excitation and emission spectra of 436 nm and 543 nm, respectively, while FITC excitation and emission are at 494 nm and 521 nm, respectively. After 48 hours of treatment of the A549 cells with 200 *μ*g/mL and 400 *μ*g/mL saffron extract, the fluorescence of the apoptotic cells was measured in the absence of PI and Annexin staining. Apoptotic cell death of saffron extract was measured using flourescein isothiocyanate (FITC)-conjugated Annexin V/PI assay kit by flow cytometry. Briefly 5 × 10^5^ cells were washed with ice-cold PBS, re-suspended in 100 *μ*L binding buffer, and stained with 5 *μ*L of FITC-conjugated Annexin V (10 mg/mL) and 10 *μ*L of PI (50 mg/mL). The cells were incubated for 15 min at room temperature in the dark, and then 400 *μ*L of binding buffer was added. After labelling, all samples were analyzed by fluorescence microscopy or analyzed by a FACScan flow cytometry (Becton-Dickinson, USA). For analysis, A549 cells were gated separately according to their granularity and size on forward scatter (FSC) versus side scatter (SSC) plot. The early and late apoptosis were evaluated on fluorescence 2 (FL2 for propidium iodide) versus fluorescence 1 (FL1 for Annexin) plots. The percentage of cells stained with Annexin V only was evaluated as early apoptosis; the percentage of cells stained with both Annexin V and propidium iodide was evaluated as late apoptosis or necrotic stage.

### 2.7. Detection of Activated Caspases in Lung Cancer Cell Line Using FLICA

FAM-VAD-FMK, a cell-permeant-fluorochrome derivate of caspase inhibitor Val-Ala-Asp-fluoromethylketone, was used to detect the activated caspases in the A549 cells. This noncytotoxic fluorescent caspase inhibitor (FLICA) binds covalently and irreversibly to many activated caspases (caspases 1, 3, 4, 5, 6, 7, 8, and 9). Therefore, it can be used as a generic probe for the detection of most caspases. The fluorogenic substrate becomes fluorescent upon cleavage by the caspases [16]. The inhibitor was used with the appropriate controls according to the instruction manual of the manufacturer (carboxyfluorescein FLICA apoptosis detection kit caspase assay, poly-caspases FLICA (FAM-VAD-FMK)). This inhibitor (FAM–VAD–FMK) which is commercially available as a component of the CaspaTag fluorescein caspase activity kit was dissolved in dimethyl sulfoxide (DMSO; Sigma) as specified in the provided protocol with the kit, to obtain 150x concentrated (stock) solution. Aliquots of this solution were stored at −20°C in the dark. Prior to use, a 30x working solution of FLICA was prepared by diluting the stock solution 1 : 5 in phosphate buffered saline (PBS) and mixing until it becomes transparent and homogeneous. Poly-caspase FLICA apoptosis detection kit contains ICT, green fluorescent-labeled inhibitor, and FAM-VAD-FMK, a potent inhibitor of caspase activity.

#### 2.7.1. Cell Staining for Analysis by Laser Scanning Cytometry (LSC)

The A549 cells from the untreated or saffron-treated cultures were centrifuged (200 ×g, 4 min) and resuspended in PBS at approximately 10^6^ cells per milliliter density. The cells were then attached electrostatically to microscope slides. The slides were then placed on the motorized stage of the LSC for fluorescence measurements (first measurement). 

#### 2.7.2. Cell Staining for Analysis by Flow Cytometry

Exponentially growing suspension cultures of the A549 cells at <5 × 10^5^ cells/mL density were treated with saffron extract at concentrations of 200 and 400 *μ*g/mL for different periods of time. The cells were then centrifuged (300 ×g, 5 min), the cell pellets (10^5^ cells) resuspended in 300 *μ*L of medium in the centrifuge tubes, and 10 *μ*L of the working solution of FAM-VAD-FMK was added to these cell suspensions. The cells were incubated for 1 h at 37°C under 5% CO_2_ and protected from the light. After the incubation, 2 mL of the working dilution of the “wash buffer” (component of the CaspaTag kit, ImmunoChemistry Technologies) was added and gently mixed. The cells were then centrifuged at 200 ×g for 5 min, the supernatant aspirated, and the cell pellet resuspended again in 2 mL of the “wash buffer” and again centrifuged as above. The cell pellet was then resuspended in 1 mL of the “wash buffer” containing 1 *μ*g/mL of PI. The samples were placed on ice and the cell fluorescence was measured during the next 15 min in the FACScan (Becton Dickinson, San Jose, CA) flow cytometer using the standard emission filters for green (FL1) and red (FL3) fluorescence photomultipliers.

A minimum of 20000 cells was examined for each assay. The cells population was gated using a 90-degree and forward-angle light scatter to exclude debris and aggregates. The selection of the area corresponding to cell was determined before hand by the analysis of purified thawed cell recovered after selection on a two-step gradient (Puresperm 90% and 45%, Nidacon International). The excitation wavelength was 488 nm supplied by an argon laser. Green (FLICA) derived fluorescence and red fluorescence (PI) were detected with FL1 (525 nm) and FL3 (620 nm) detections. FL1 and FL3 fluorescence signals were recorded after logarithmic amplification and the rates of stained cells were automatically computed by the flow cytometer (Coulter, Villepinte, France). For a bicolour analysis, four types of samples were measured to set up electronic compensation and quadrant statistics unstained A549 cells (FLICA replaced by PBS), the A549 cells stained with FLICA, the A549 cells stained with PI, and the A549 cells stained with PI and FLICA (Figure 5).

#### 2.7.3. Cell Staining for Analysis by Flourescent Microscope

The A549 cells were attached electrostatically to microscope slides in 6-well plates and allowed to attach for 24 h to keep the log-phase growth at the time of drug treatment. Saffron at different concentrations was added to the wells for 48 hours. After the treatment with saffron for 48 h, the media were removed and 10 *μ*L of FLICA working solution was added into 300 *μ*L of culture medium. After 1 h incubation at 37°C, the staining solution was then removed by vacuum suction and the cells were rinsed with PBS, and 1 *μ*L Hoechst was added into culture medium and incubated for 5 minutes. The cells were rinsed by 2 mL of 1x wash buffer, and one drop of this buffer was split on a lamella, and cover slips were put on it and were then observed by florescent microscope.

For fluorescence microscopy, the analysis of the sample was performed by conventional epifluorescent microscopy (excitation: 450–490 nm; emission: 525–617 nm). Carboxyfluorescein (FAM-VAD-FMK) of the FLICA was observed as green-colored and PI as red-colored fluorescence. A minimum of four-hundred cells was randomly assessed per slide in at least five fields. Four patterns of fluorescence were measured (Figure 7).

1. Viable cells without staining of activated poly-caspases: Casp−/PI− (only observed with bright light microscopy).
2. Dead cells without staining of activated poly-caspases: Casp−/PI+ (red).
3. Viable cells with staining of activated poly-caspases (early apoptotic cells): Casp+/PI− (green).
4. Dead cells with staining of activated poly-caspases (late apoptotic cells) Casp+/PI+ (red and green).

### 2.8. Statistical Analysis

 All results were expressed as mean ± SEM. The significance of difference was evaluated with ANOVA and Bonferroni test. A probability level of *P* < 0.05 was considered statistically significant.

## 3. Results

### 3.1. Effects of Aqueous Extract of Saffron on Cell Viability

In order to evaluate the effect of aqueous extract of saffron on growth of the MRC-5 cells, normal cells, and the A549 cells, human lung cancer cells, the cells were treated with different concentrations of saffron for 3 days and their growth inhibitory effects were compared. The impact of aqueous extract of saffron on cell viability was quantitated by MTT assay. Aqueous extract of saffron showed significantly high growth inhibitory effects on A549 cell line in a dose-dependent manner (*P* < 0.001) compared to the MRC-5 cells. Aqueous extract of saffron (200, 400, and 800 *μ*g/mL) decreased cell viability in malignant cells but not in nonmalignant cells after 24 h (*P* < 0.05, *P* < 0.01, and *P* < 0.001, resp.) (Figure 1). This toxicity was consistent with morphologic changes. However, the extract at different concentrations could not decrease cell viability in the MRC-5 cells. After 48 h, even low dose of extract (100 *μ*g/mL) decreased cell viability in lung cancer cells (*P* < 0.05), and higher concentrations of aqueous extract of saffron (400, 800 *μ*g/mL) dramatically decreased cell viability in A549 cells compared to the MRC-5 cells (*P* < 0.001) (Figure 1(b)). After 72 h, again aqueous extract statistically deceased cell viability in the A549 cells in comparison with the MRC-5 cells even at lower concentration (100 *μ*g/mL) (Figure 1(c)). The dose inducing 50% cell growth inhibition (IC_50_) against A549 cells was 380 ± 9.6 and 170 ± 2.5 *μ*g/mL after 48 and 72 h, respectively (Table 1). 

### 3.2. Morphological Evaluation

Morphological studies were carried out to observe the morphological changes of cell death on the A549 cells elicited by the saffron extract. As shown in Figure 2, after 48 h of incubation with concentrations of 200 and 400 *μ*g/mL of aqueous extract of saffron, morphological changes were observed using the normal inverted microscope in comparison with the control which is consisting of reduction in number of living cells, volume, and rounding until the nucleus constituted the majority of the cellular volume. No significantly morphological changes were detected in MRC-5 cells (data was not shown). In Figure 2(a) (control), the cells were incubated in drug-free medium for 48 h. As clearly shown in Figure 2(b), the aqueous extract (200 *μ*g/mL) inhibited the growth of the A549 cells after 48 h in comparison with the control (Figure 2(a)); however, Figure 2(c) shows that the treated cells with the higher dose of saffron aqueous extract (400 *μ*g/mL) had more prominent growth inhibition and shrinkage of the cells compared with treated cell with a lower dose of saffron (200 *μ*g/mL) which consisted of induction in number of living cells, volume, and rounding and confirmed our MTT results.

### 3.3. Quantification Studies for Apoptosis by Saffron Extract

To study roles of aqueous extract of saffron in apoptosis, saffron extract was used to set up apoptosis system on A549 cell line. The A549 cells were treated with concentrations of 200 and 400 *μ*g/mL saffron extract for 48 h. After treatment, the cells were harvested, and apoptosis was examined by flow cytometry (Figure 3). Quantitative analysis using Annexin V/PI assay further showed that the proportion of the early stage apoptotic cells (Annexin V+/PI−) increased significantly from 14.50% to 37.5%, while proportion of the late stage apoptotic cell (Annexin V+/PI+) increased significantly from 18.50% to 46.5% when the cells were treated with the concentrations of 200 and 400 *μ*g/mL aqueous extract of saffron, respectively (Figure 4). Apoptosis induced from 200 and 400 *μ*g/mL of saffron extract was statistically higher than control, and the percentage of the early and late apoptotic cells significantly increased by increasing saffron concentration (*P* < 0.001). 

### 3.4. Effect of Aqueous Extract of Saffron on Caspase Activity

To further confirm the apoptotic activity of saffron extract to activate to the effector caspase was determined using a potent fluorescent-labeled caspase inhibitor that covalently binds to active caspase within the cells. 

Four cell subpopulations representing nonapoptotic cells at three consecutive stages of apoptosis were distinguished on the bivariate distributions (scatterplots) representing green versus red fluorescence of the cells stained with FAM-VAD-FMK and PI (Figure 5). To determine whether caspases play a role in saffron-extract-mediated apoptosis of the A549 cells, we assessed the activated caspases by using carboxyfluorescein FLICA poly-caspases technique after treatment with different concentration of saffron using flow cytometry (FCM) and fluorescent microscope. As shown in Figure 5(A), the unlabeled cells, which have neither green nor red fluorescence, are nonapoptotic cells (Figure 5(a); left bottom quadrant). The cells that have only green fluorescence are early apoptotic cells; they exclude PI but have already activated caspases (Figure 5(b); left top quadrant). More advanced in apoptosis are the cells with the compromised plasma membrane that bind FAM-VAD-FMK and stain with PI (Figure 5(c); right top quadrant). At the final stage of apoptosis, the cells stain with PI but do not demonstrate active caspases (Figure 5(d); right bottom quadrant). The cells of the last two subpopulations, unable to exclude PI, represent the necrotic stage of apoptosis (secondary necrosis). 

Analysis of the scatterplots of the cells exposed to aqueous extract of saffron reveals that saffron-induced apoptogenic effects. The distributions of the A549 cells exposed to aqueous extract of saffron concentrations (200 and 400 *μ*g/mL) for 48 h were different to those of untreated control cells (Figures 5(B) and 5(C), resp.). The percentages of cells in the subpopulations (“b” and “c” shown in the respective quadrants in Figures 5(B) and 5(C)) in saffron-treated cultures were significantly increased as opposed to the untreated cultures (Figure 5(A)). As shown in Figures 5(B) and 5(C), the direct transition from FLICA−/PI− to FLICA−/PI+ (from quadrant “a” to “ c”), by passing the FLICA+ stages (quadrant “b”) in treated groups, may be considered as the marker of a primary cell necrosis and the evidence of presence of activated caspases. But the loss of cells' ability to bind FLICA at the late stage of apoptosis indicates that caspases are either inactivated, degraded, or excreted at that time point. Hence, the late apoptotic cells may not be identified solely on the evidence of the presence of activated caspases. In the A549 cells, it can be inferred that apoptosis involves caspase signaling since, at least, some of the caspases 1, 3, 4, 5, 6, 7, 8, and 9 were found to be activated by saffron.

### 3.5. Aqueous Extract of Saffron Induces Activation of Caspase Pathway

To determine whether caspase plays a role in saffron-extract-mediated apoptosis of the A549 cells, we assessed the activated caspases 1, 3, 4, 5, 6, 7, and 9 protein level of the A549 cells with and without treatment with saffron extract using flow cytometry (FCM). As shown in Figure 6, after 48 h of the A549 cells being exposed to saffron extract for different concentrations (200 and 400 *μ*g/mL), the percentage of activated caspases 1, 3, 5, 6, 7, 8, and 9 increased from 2.4%, to 25.7%, 61.5%, respectively. These findings suggest that the mechanism of the A549 cells apoptosis induced by saffron extract is involved in activation of caspases. Fluorescein was measured on the FL1 channel and a log FL1 (*x*-axis) versus number of cells (*y*-axis) histogram may be generated. On this histogram, there appeared two cell populations represented by two peaks. The majority of the caspases negative cells occurred within the first log decade of the FL1 (*x*) axis (first peak), whereas the caspase-positive cell population appeared as a separate peak or as a shoulder of the first peak showing increased fluorescence intensity. The cells with the active caspase (those undergoing apoptosis) fluoresce green. In Figure 6, the A549 cells were treated with media, noninduced cells, Figure 6(a) or saffron 200 *μ*g/mL Figure 6(b) or 400 *μ*g/mL Figure 6(c), induced cells, for 48 hours. The frequency histogram of the number of events (*Y* axis) versus fluorescein intensity (*X* axis) showed 2 peaks: caspase-negative cells occur to the left of the M1 region (unlabeled cells, Figure 6(a)); caspase-positive cells lay within the M1 region (cells were labeled with FLICA, Figures 6(b) and 6(c)). Figure 6, showed that the nontreated cells had 2.4% caspase-positive cells and 97.6% caspase-negative cells, while the cells treated with different saffron extract concentrations (200 and 400 *μ*g/mL) had 25.7 and 61.5% caspase-positive cells, respectively. These findings suggest that the mechanism of the A549 cell apoptosis induced by saffron extract is involved in activation of some of the caspase pathways.

### 3.6. Fluorescence Microscopy for Adherent A549 Cells

To further define the role of caspase in saffron extract-induced apoptosis, cells were treated with broad-spectrum caspase inhibitor, the FAM-VAD-FMK. Then, the cells were assessed by fluorescence microscopy. Viewing cells through a fluorescence microscope, apoptotic cells showed fluorescence greens, while nonapoptotic cells appeared mostly unstained. All the cells were stained with Hoechst. As apoptosis progresses (treatment of the cells with increasing concentrations of saffron from 200 to 400 *μ*g/mL), the amount of active caspase enzymes capable of binding the labeled inhibitor increased. Therefore, our results indicated that the treated A549 cells (400 *μ*g/mL) in more advanced stages of apoptosis appeared brighter green than the treated cells (200 *μ*g/mL) in earlier stages (Figure 7). In Figure 7, A549 cells in Figure 7(a) (which were not visible in photo Figures 7(b) and 7(c)) did not have a brightly stained nucleus; therefore, the cells were not apoptotic nor necrotic. The cells (Figure 7(a)) photographed under a different wavelength for Hoechst stain, appear blue. It means that these cells did not bind to the reagent and therefore are not apoptotic.  Figure 7(b) showed that few cells had very brightly stained nucleus (arrows)—their DNAs were condensing in the cells, a sign they were dying and also somewhat appeared green—they were apoptotic and stained positive for poly-caspases activity with the FAM-VAD-FMK reagent. The other cells, which did not have brightly stained nucleus, did not bind to the reagent and therefore were not apoptotic. This cell did not stain green so it is either necrotic (caspases were not activated and therefore could not bind to FAM-VAD-FMK) or apoptotic but far past the active caspase stage and therefore did not stain green with FAM-VAD-FMK because the caspases were no longer active. The cells (Figure 7(c)) which appear green, in some cells, had very brightly stained blue nucleus (spots), indicating that chromosome condensation had begun and the cells were beginning to die and there were cells that appeared green. They were apoptotic and stained positive for poly-caspases activity with the FAM-VAD-FMK reagent. They also had many bright blue spots from the Hoechst stain, indicating that the cell is beginning to die.

## 4. Discussion

Establishment of effective therapies for lung cancer is a major concern in clinical cancer research. Although there are an increasing number of therapeutic options available for patients with cancer, their efficacy is time-limited and noncurative. Selective activation of apoptosis is often cited as one of the major goals of cancer chemotherapy. It is currently thought that dysregulated cell cycle proliferation and apoptosis are important factors in the development of cancer [17]. Therefore, it appears that exploiting the apoptotic potential of cancer cells might lead to new therapies that could be less toxic to normal cells due to the physiologically controlled survival pathway [18].

Approximately 50–60% of cancer patients in the United States utilize agents derived from different parts of plants or nutrients (complementary and alternative medicine), exclusively or concurrently with traditional therapeutic regime such as chemotherapy and/or radiation therapy. The need for new drugs has prompted studies evaluating possible anticancer agents in fruits, vegetables, herbs, and spices. Saffron, a spice and a food colorant present in the dry stigmas of the plant *Crocus sativus* L., has been used as an herbal remedy for various ailments including cancer by the ancient Arabian, Indian, and Chinese cultures. Saffron has been shown to exhibit good antioxidant and anticancer activity. The present study was initiated with the purpose of evaluating the action of saffron on the adenocarcinomic human alveolar basal epithelial cells. The rationale for this study was on the basis of several data that linked saffron to the treatment of various diseases [6, 9], together with the favorable antitumoral action of saffron recently [19, 20].

The experimental results show that saffron had good cytotoxicity against the A549 cells but was less sensitive to normal human cells, including the normal human lung fibroblast cell (MRC-5), based on the high IC_50_ value (Table 1). The high sensitivity of the malignant cells may in part reflect the difference in growth rates between the malignant and nonmalignant cells. Experimental results imply that the cytotoxic behavior of saffron toward the A549 cells was selective. Saffron treatment inhibited the A549 cell growth in a dose- and time-dependent manner (Figure 1). The highest cytotoxicity on the A549 cells occurred at 72 h (Figure 1(c)), indicating that saffron has a long-term effect. Based on morphological changes identified by inverse microscopy, typical morphological characteristics of apoptosis and the reduction of the cells were observed (Figure 2). Based on the facts that saffron showed significant antitumor effects against tumor cells, attempts were made to examine its antitumor activities and possible involved mechanisms against the human lung adenocarcinoma epithelial cells. 

The present study found that saffron can induce apoptosis and active caspases in the A549 cells. It is likely that the anti-proliferative effect of saffron on the lung cancer cells is due to growth inhibition of cells induced by apoptosis. To the authors' knowledge, this is the first report on saffron-induced cytotoxicity activity and apoptosis through caspase pathways in human alveolar basal epithelial cells. 

Our results using Annexin V-FITC/PI labelling indicated that saffron could induce apoptosis in a time-dependent manner. It suggests that the growth inhibition of saffron for the A549 cells is caused by apoptosis [20–22]. Generally, apoptosis can occur via two fundamental pathways: (1) the mitochondrial or intrinsic pathway and (2) the death receptor or extrinsic pathway [23]. The intrinsic pathway is triggered by release of mitochondrial proteins, such as cytochrome c, which bind with Apaf-1 and procaspase-9 in a dATP-dependent manner to form the apoptosome [24]. The apoptosome can induce activation of caspase-9, thereby initiating apoptotic caspase cascades [25, 26]. Conversely, the extrinsic pathway is initiated by the interaction of ligands with their respective death receptors, sequentially leading to cleavage of initiator caspase-8. The active caspase-8 cleaves executioner caspase-3, resulting in apoptosis [27]. The apical proteases in the intrinsic and extrinsic pathways are caspase-9 and caspase-8, respectively. Activated caspase-9 and caspase-8 further initiate activation of the caspase cascade, leading to biochemical and morphological changes associated with apoptosis [28, 29]. Caspase-3 is a well-known downstream adaptor caspase which can be proteolytically activated by caspase-9 or caspase-8 via mitochondrial or cell death receptor signaling pathways [30–32]. Thus, caspases have been shown to be activated during apoptosis in many cells and play critical roles in both initiation and execution of apoptosis [33]. Sharma et al. (2009) reported that tumors arise more frequently through, intrinsic pathway than the extrinsic pathway because of the sensitivity [34].

To investigate the mechanism of cell death induced by saffron in the A549 cells, flow cytometric analysis was done by PI and Annexin V-FITC labeling to confirm apoptosis/necrosis as a marker to assess apoptosis [18]. The results of the present study indicated an increase in apoptotic population induced by saffron in a concentration-dependent manner. The mechanism of action of saffron on lung cancer cells is likely complex but the current result showed at least a partial involvement apoptosis. Therefore, our results indicate that apoptotic cell death may play a role in the action of saffron on lung cancer cells. This opens the interesting possibility of using therapies that control cell growth in cancer tissues of the lung that may prevent metastases. The early apoptotic cells tend to exhibit phosphatidylserine on outer cell membrane, which is normally positioned across the inner membrane [35] and it has a strong binding affinity to annexin V [36]. Determination of exposure of phosphatidylserine on the cell surface as an early event in the A549 cells treated with saffron was confirmed by annexin V-FITC/PI (Figures 6 and 7). It is well established that agents that are capable of inducing apoptosis as mode of cell death are good anticancer candidates [37]. Therefore, saffron is potential anticancer candidates that are believed to possess the characteristics of inducing apoptosis selectively in cancer cells.

Following this reasoning, we studied the possible molecular mechanism that is involved in apoptotic effects of saffron on A549 cell line. With respect to the mechanism of the action of saffron on the A549 cell apoptosis, our studies indicated that saffron exerted a higher effect on the levels of caspase pathways. It is possible that changes in the levels of caspase may play a role in the action of saffron treatment on these cells. 

Although the precise molecular mechanisms of cytotoxic activities of saffron are still ambiguous, the recent finding that caspase pathway is a molecular target of saffron [38] encourages further study of saffron compounds.

Activation of the family of caspases was known as a crucial mechanism for induction of death signals to apoptosis. Caspases participate in a cascade that is triggered in response to proapoptotic signals and culminates in cleavage of a set of proteins, resulting in disassembly of the cell [39, 40]. The family of caspase is the primary activator of apoptotic DNA fragmentation [41–43]. Our results showed that saffron can cause activation, some of caspases 1, 3, 4, 5, 6, 7, 8, and 9 in a time-dependent manner, but not necessarily all of them. Elevation of caspases by saffron was initiated after 24 h of saffron exposure and maintained at least for 48 h. It indicates that saffron-induced apoptosis is mediated by caspase-dependent pathways. A recent finding further supports this suggestion as the parent compound and rographolide were shown to have novel mechanisms of antitumor activity by targeting the cascade caspases through increasing the caspases 1, 3, 5, 7, and 9 signalling pathway [38]. It has recently been demonstrated that FLICA covalently binds to a larger subunit of active caspases produced by proteolytic cleavage of the proenzyme [44, 45]. Therefore, the FLICA assay is fit for the poly-caspases analysis, but it would be prudent to support this test with other specific methods for the detection of activated caspases, such as western blot analysis and measurement of caspases activity. 

## 5. Conclusions

The findings of our study have important clinical implications. These results demonstrate the potential anticancer activity of saffron against the carcinomic human alveolar basal epithelial cell. Saffron exhibited a strong inhibitory effect on the proliferation of the A549 cells in vitro. The anticancer activity of saffron could be attributed in part to its inhibition of proliferation and apoptosis induction of cancer cells through causing caspases activation. 

Altogether, the present study shows toxicity of saffron in the A549 cell line with involvement of apoptosis or programmed cell death through causing caspase pathways. Further studies are needed to fully recognize the mechanisms involved in cell death by saffron and variety of biologically active ingredients isolated. Saffron could also be considered as a promising chemotherapeutic agent in treatment of lung cancer.

## Figures and Tables

**Figure 1:** Exposure of the A549 cells for 24, 48, and 72 h with saffron. Cells were treated with different concentrations of saffron extract (100, 200, 400, and 800 *μ*g/mL) for 24 (a), 48 (b), and 72 (c) hours. Viability was quantitated by MTT assay. Results are mean ± SEM. The asterisks are indicators of statistical difference obtained separately at different time points compared to their controls shown in figure as *P < 0.05, **P < 0.01, and ***P < 0.001.

**Figure 2:** Comparison of cytotoxicty effect of saffron on cell viability of the A549 cells. Morphological changes of cells after 48-hour treatment with different concentrations of saffron (200, 400 *μ*g/mL), (a) untreated A549 cells (b) the A549 cells treated with 200 (*μ*g/mL) saffron and (c) the A549 cells treated with 400 (*μ*g/mL) saffron.

**Figure 3:** Assessment of apoptosis by Annexin V/PI on the alveolar human lung cancer cell line (A549). The cells were treated with 200 and 400 *μ*g/mL saffron extract for 48 h (symbols (b), (c)) or media (control symbol (a)), and apoptosis was examined with flow cytometry after Annexin V-PI double staining. The necrotic cells lost cell membrane integrity that permits PI entry. Viable cells exhibit Annexin V (−)/PI (−) (symbol (a)); early apoptotic cells exhibit Annexin V (+)/PI (−) (symbol (b)); late apoptotic cells or necrotic cells exhibit Annexin V (+)/PI (+) (symbol (c)).

**Figure 4:** Assessment of apoptosis by Annexin V/PI on alveolar human lung cancer cell line (A549 cells). Percentage of cell death based on the assessment of apoptosis by Annexin V/PI. ***, ^###^ *P* < 0.001 compared with control and the other dose, respectively.

**Figure 5:** Effect of saffron on exponentially growing A549 cells. Scattergrams of LSC measurements representing the cells stained with FAM-VAD-FMK (green fluorescence) and PI (red fluorescence). (A) Control cells exponentially growing in standard condition. (B) Cells exposed to 200 *μ*g/mL saffron for 48 h during exponential growth. (C) Cells exposed to 400 *μ*g/mL saffron for 48 h during exponential growth. Each scatterplot is divided into four compartments depending on the cell status as revealed by green versus red fluorescence. a: live cells; b: early apoptotic cells; c: late apoptotic cells; d: secondary necrotic cells.

**Figure 6:** The A549 cells were treated with media, noninduced cells (a) or saffron extract 200 *μ*g/mL (b) or 400 *μ*g/mL (c) induced cells, for 48 hours. Cells were labeled with FAMVAD-FMK for 1 hour, washed, and analyzed. Caspase activity was detected using a BD FACSCalibur flow cytometer.

**Figure 7:** Nuclear changes of saffron-treated A549 cells. A549 cells seeded on chamber slides were treated with media or different saffron concentrations. Suspension of the A549 cells was incubated with media (a), 200 *μ*g/mL of saffron (b), and 400 *μ*g/mL of saffron (c) for 48 hours at 37°C to induce apoptosis. Cells were then labeled with FAM-VAD-FMK for 60 minutes at 37°C. Cells were washed, and then Hoechst stain was added and incubated for 5 minutes. Wet-mount slides were prepared and the photos of the same cells were taken and superimposed. Caspase activity (green) was detected using a band pass filter (excitation at 488 nm, emission at 520 nm). Nuclear staining by Hoechst stain (blue) was revealed using a UV filter (excitation at 365 nm, emission at 480 nm). In these pictures, the yellow arrows represent the nuclear breakdown and chromatin condensation of A549 cells induced by saffron.

**Table 1:** Doses inducing 50% cell growth inhibition (IC_50_) of aqueous extract of Saffron against lung cancer cell line (A549).

IC_50_	48 h	72 h

A549	380 ± 9.6	170 ± 2.5

Cells were treated with different concentration of Saffron for 24, 48 and 72 hours. Viability was quantitated by MTT assay.
